# The Quantity and Quality of Lumbar Muscles and Lumbopelvic Parameters in Patients With Degenerative Spondylolisthesis

**DOI:** 10.7759/cureus.18428

**Published:** 2021-10-01

**Authors:** Shuhei Ohyama, Yasuchika Aoki, Masahiro Inoue, Takayuki Nakajima, Yusuke Sato, Hiroyuki Fukuchi, Takayuki Sakai, Shigehiro Ochi, Noriyuki Yanagawa, Seiji Ohtori

**Affiliations:** 1 Department of Orthopaedic Surgery, Eastern Chiba Medical Center, Togane, JPN; 2 Department of Radiology, Eastern Chiba Medical Center, Togane, JPN; 3 Department of Orthopaedics, Chiba University Hospital, Chiba, JPN; 4 Department of Orthopaedic Surgery, Graduate School of Medicine, Chiba University, Chiba, JPN

**Keywords:** fat infiltration, cross-sectional area, lumbar lordosis, lumbopelvic parameters, lumbar muscle, degenerative spondylolisthesis

## Abstract

Introduction

Lumbar degenerative spondylolisthesis (DS) is one of the most common causes of low back pain. The lumbar muscles, such as the psoas major (PM), erector spinae (ES), and multifidus (MF) muscles, play an important role in the stability and functional movement of the lumbar spine. The quantities and qualities of these muscles may be related to the occurrence of DS and lumbopelvic parameters, such as lumbar lordosis (LL) and sacral slope (SS). However,the influence of lumbar muscles on DS and lumbopelvic alignment is not well understood.

Methods

Patients with L4 DS (DS group, n=25) and without DS (non-DS group, n=25) were included. Using sagittal reconstructed CT images of patients who visited our hospital for reasons other than low back disorders, LL, upper lumbar lordosis ([ULL] L1-L4), lower lumbar lordosis ([LLL] L4-S1), and SS were examined. To evaluate the quantity and quality of lumbar muscles, the gross cross-sectional area (GCSA), functional cross-sectional area (FCSA), and fat infiltration (FI) of the PM, ES, and MF muscles were measured by CT images. The lumbopelvic parameters, FCSA, GCSA, and FI of lumbar muscles were compared between the two groups. Then, each lumbar muscle parameter was analyzed for correlation with DS and lumbopelvic parameters.

Results

DS patients displayed significantly greater ULL and lower FI of the PM and ES muscles than non-DS patients (p=0.0078, 0.031, and 0.010, respectively). The FI of the ES muscle was significantly correlated with the presence of DS (p=0.010). The FCSA of the ES and MF muscles and the GCSA of the MF muscle showed a significant correlation with LL and SS in the non-DS group (p<0.05), but not in the DS group..

Conclusion

ULL was greater in L4 DS patients, possibly related to the better quality of the ES muscle. All DS patients showed mild (grade I) spondylolisthesis, suggesting the possibility that lumbar muscle quality is better in patients with mild DS than in those without DS. The ES and MF muscles may play an important role in maintaining the lumbar lordotic angle in non-DS patients but not in DS patients.

## Introduction

Degenerative spondylolisthesis (DS) is a disorder that causes the slip of one vertebral body over the one below (usually L4 on L5). It differs from isthmic spondylolisthesis (IS) in terms of the absence of a pars interarticularis defect (spondylolysis) [1]. DS is one of the most common causes of low back pain (LBP) [2].

The lumbar muscles, such as the psoas major (PM), erector spinae (ES), and multifidus (MF) muscles, play an important role in the stability and functional movement of the lumbar spine. To evaluate the quantity of the lumbar muscles, the cross-sectional area (CSA) is measured by computed tomography (CT) or magnetic resonance imaging (MRI), both of which are recognized as reliable methods for the evaluation of CSA of lumbar muscles [3,4]. The measurement of the functional cross-sectional area (FCSA), i.e., the area of lean muscle tissue within a muscle’s fascial boundaries, is a better indicator of the muscle’s contractile ability [5]. To evaluate the quality of the lumbar muscles, fat infiltration (FI), CT and MRI are commonly utilized. Although MRI is more commonly used, several previous studies have used CT for the evaluation of FI and reported the reliability of CT evaluation [6-9]. The CSA and FI of the lumbar muscles are associated with age, sex, body mass index (BMI), and LBP [10-12]. In a previous study, the FI could be measured as the ratio of FCSA to gross cross-sectional area (GCSA) [13].

The importance of sagittal alignment in the treatment of patients with adult spinal deformities has been widely recognized [14,15]. Radiographs taken in the standing position are usually used for the evaluation of lumbopelvic alignment. However, several recent studies used CT images in the supine position for the evaluation of lumbopelvic parameters [16,17]. Based on these observations, CT images were utilized in the present study for the analysis of the lumbar spine in patients who visited our hospital for reasons other than low back disorders.

We found that in patients with IS, atrophy of the PM is more significantly correlated with the progression of vertebral slip and greater lumbar lordosis (LL) and sacral slope (SS) than in patients without IS [18].

The association between DS and lumbar muscles (CSA and FI) is not well understood. A previous study reported that there is no correlation; however, another study reported that there is an association between MF atrophy and DS [19,20]. Therefore, this study aimed to elucidate the association among DS, lumbar muscles, and lumbopelvic parameters by performing CT imaging and analysis for correlations.

## Materials and methods

Patients

Consecutive patients who underwent CT scans of the abdominal or lumbar regions for reasons other than low back disorders between July 2015 and February 2016 were included in the study. Patients with prevalent vertebral fractures between the T10 and L5 levels, previous lumbar spinal fusion surgery, and bilateral and unilateral spondylolysis were excluded. Finally, CT images of 545 patients who met the criteria were then used for the data analysis.

The patients’ age and sex were analyzed, and sagittal multiplanar reconstructed CT images were obtained. First, the presence of L4 spondylolisthesis was examined. The data of patients with DS were also reviewed. DS was defined as the presence of vertebral slip (>3 mm), and the degree of vertebral slip was evaluated using the Meyerding grading system (grade I: <25%; grade II: 25%-50%; grade III: 50%-75%; and grade IV: 75%-100%).

The patients were divided into two groups. The first group (DS group) consisted of patients with L4 DS. For the second group (non-DS group), patients were extracted from patients without vertebral slip at any lumbar levels who were matched for age and sex with the DS group, using propensity score matching with a tolerance of 0.01. Propensity score matching was performed using the software Easy R (EZR, Saitama Medical Center, Jichi Medical University, Saitama, Japan). Using coronal reconstructed CT images, the presence of scoliosis (≥10°) at levels between T10 and S1 was examined in both groups.

Ethical considerations

The study was carried out in accordance with the Declaration of Helsinki, and the study protocol was approved by the Institutional Review Board of our medical center. All patients provided informed consent for the future use of clinical information, including CT images, and were given the opportunity to opt out of the study at any time.

Measurement of sagittal lumbopelvic parameters

Using sagittal reconstructed CT images, LL (angle between the superior endplates of L1 and S1), upper lumbar lordosis ([ULL] angle between the superior endplates of L1 and L4), lower lumbar lordosis ([LLL] angle between the superior endplates of L4 and S1), and SS (angle between the superior endplate of S1 and the horizontal plane) were examined in both groups (Figure 1).

**Figure 1:** Measurement of sagittal lumbopelvic parameters (A) Using sagittal reconstructed CT images, lumbar lordosis ([LL] angle between the superior endplates of L1 and S1), upper lumbar lordosis ([ULL] angle between the superior endplates of L1 and L4), and lower lumbar lordosis ([LLL] angle between the superior endplates of L4 and S1) were examined. (B) The sacral slope ([SS] angle between the superior endplate of S1 and the horizontal plane) was also examined.

Measurement of FCSA, GCSA, and FI of the PM, ES, and MF muscles

Using reconstructed CT images for the disc level at L4-L5 parallel to the inferior endplate of L4, measurement of the FCSA and GCSA of the PM, ES (the iliocostalis lumborum and longissimus iliocostalis), and MF muscles was performed for both groups. The measurements were obtained using the ZIO station 2 workstation software (Ziosoft, Tokyo, Japan). The FCSA was defined as the area of lean muscle tissue within the fascial boundaries of the muscle. The GCSA was defined as the area within the fascial boundaries of the muscles. To determine the lean muscle FCSA (in cm^2^), the region of interest (ROI) was drawn around the muscles of interest, carefully avoiding nearby fat, bony structures, and other soft tissues (Figure 2). To determine the GCSA (in cm^2^), the ROI was drawn around the outer perimeter of the muscle to include any areas of intramuscular fat (Figure 2). To decrease the bias caused by the differences in individual body size, the total FCSA and GCSA of the bilateral PM, ES, and MF muscles were divided by the vertebral body CSA at the middle level of the L4 pedicle (muscle CSA/vertebral body CSA) to represent the lumbar muscle FCSA and GCSA index in each individual. Patients with DS often show intervertebral disc bulging and degenerative changes of the lower endplate, such as osteophytes. To evaluate the accuracy of the CSA, the measurements of this level were selected. To determine the vertebral body CSA, the ROI was drawn around the vertebral body, cautiously avoiding osteophytes (Figure 3). The FI was calculated using the FCSA and GCSA: FI = (GCSA - FCSA) / GCSA.

**Figure 2:** Measurement of the functional cross-sectional area and gross cross-sectional area of the lumbar muscles (A) Axial reconstructed CT images. Measurements of the functional cross-sectional area of the right-side PM, ES, and MF muscles are shown. Measurements of the gross cross-sectional area of the left-side PM, ES, and MF muscles are shown. (B) Sagittal reconstructed CT images showing L4 degenerative spondylolisthesis. The level from which measurements are taken (white arrow) was the disc level at L4-L5 parallel to the inferior endplate of L4 (white dotted line). PM, psoas major; ES, erector spinae; MF, multifidus; L, left; R, right

**Figure 3:** Measurement of the vertebral body cross-sectional area (A) Axial reconstructed CT images. Measurements of the cross-sectional area of the vertebral body (VB) are shown. (B and C) Sagittal reconstructed CT images showing the level from which measurements are taken: at the middle level of the L4 pedicle (white dotted line).

Comparison of demographic data, degree of slip, scoliosis, and lumbopelvic parameters between the DS and non-DS groups

For both groups, the demographic data (sex and age), degree of slip, scoliosis, and lumbopelvic parameters (LL, ULL, LLL, and SS) were compared. We calculated the mean values and standard deviations (SDs).

Comparison of the FCSA index, GCSA index, and FI of lumbar muscles between the DS and non-DS groups

For both groups, the FCSA index, GCSA index, FI of the lumbar muscles (PM, MF, and ES), and L4 vertebral body CSA were compared. The mean values and SDs were calculated for each group.

Correlation between the FCSA index, GCSA index, and FI of lumbar muscles, and DS

Multiple regression analysis was performed to evaluate for correlations between the FCSA index, GCSA index, and FI of lumbar muscles, which showed significant differences between both groups, and DS after adjustment for age, sex, scoliosis, and lumbopelvic parameters (LL and SS).

Correlation between the FCSA index, GCSA index, FI of lumbar muscles, LL, and SS, and scoliosis

Multiple regression analysis was performed to evaluate for correlations between the FCSA index, GCSA index, FI of lumbar muscles, LL, and SS, and scoliosis after adjustment for age and sex.

Correlation between the FCSA index, GCSA index, and FI of lumbar muscles, and the lumbopelvic parameters in each group

Simple regression analyses were performed to evaluate for correlations between the FCSA index, GCSA index, or FI of lumbar muscles, and the lumbopelvic parameters (LL and SS).

Data analysis

To compare the age, lumbopelvic parameters, FCSA index, GCSA index, and FI of lumbar muscles between both groups, an unpaired t-test was used. A χ2 test was employed to compare sex and the presence of scoliosis. To investigate the correlation between the FCSA index, GCSA index, or FI of lumbar muscles, and DS, a multiple regression analysis was performed after appropriate adjustment for age, sex, scoliosis, and lumbopelvic parameters (LL and SS). To investigate the correlation between the FCSA index, GCSA index, FI of lumbar muscles, and lumbopelvic parameters (LL and SS), and the presence of scoliosis, a multiple regression analysis was performed after appropriate adjustment for age and sex. To investigate the correlation between the FCSA index, GCSA index, or FI of lumbar muscles, and the lumbopelvic parameters (LL and SS), a simple regression analysis was used. Statistical significance was set at p<0.05. Values are expressed as mean ± SD.

## Results

Differences in demographic data, degree of slip, scoliosis, and lumbopelvic parameters between the DS and non-DS groups

This study included 708 consecutive patients. In total, 127 patients with prevalent vertebral fractures between the T10 and L5 levels or previous lumbar spinal fusion surgery were excluded; 36 patients with spondylolysis were also excluded from the study. After exclusion, a total of 545 patients were enrolled in the study. Of the patients, 25 (mean age: 74.7±9.3 years; 13 males/12 females) had L4 DS (DS group, Table 1). Another 25 patients (mean age: 74.7±9.3 years old; 13 males/12 females) without DS were age- and sex-matched using propensity score matching (non-DS group, Table 1). The degree of vertebral slip in all patients in the DS group was classified as grade I. One patient in the DS group and five patients in the non-DS group had scoliosis.

**Table 1:** Demographic data, scoliosis, and lumbopelvic parameters in the DS group and the non-DS group Data are presented as mean ± standard deviation. Asterisk (*) indicates statistically significant differences (p<0.05).

	DS	Non-DS	p-Value
Number of patients	25	25	1.0
Age (years)	74.5±9.3	74.5±9.3	1.0
Sex (male/female)	13/12	13/12	1.0
% scoliosis	4% (1/25)	20% (5/25)	0.082
Lumbopelvic parameters (°)			
LL	44.9±10.3	39.1±11.8	0.075
ULL	18.9±6.8	11.8±10.4	0.0078*
LLL	26.0±3.4	27.4±1.4	0.61
SS	39.6±8.5	37.0±8.5	0.30
DS, degenerative spondylolisthesis; non-DS, non-degenerative spondylolisthesis; LL, lumbar lordosis; ULL, upper lumbar lordosis (angle between the superior endplates of L1 and L4); LLL, lower lumbar lordosis (angle between the superior endplates of L4 and S1); SS, sacral slope			

The DS group showed a trend toward greater LL (44.9±10.3°) than the non-DS group (39.1±11.8°). However, there were no significant differences in LL (p=0.075). ULL was significantly greater in the DS group (18.9±6.8°) than in the non-DS group (11.8±10.4°) (p=0.0078, Table 1). LLL did not differ between the two groups. There were no significant differences in SS between the DS group (39.6±8.5°) and the non-DS group (37.0±8.5°) (Table 1).

Differences in the FCSA index, GCSA index, and FI of lumbar muscles between the DS and non-DS groups

In terms of the FCSA index, there were no significant differences in the PM, ES, and MF muscles between the DS group (PM, 1.3±0.3; ES, 1.4±0.3; MF, 0.7±0.2) and the non-DS group (PM, 1.2±0.3; ES, 1.2±0.4; MF, 0.8±0.2) (Table 2). With regard to the GCSA index, there were no significant differences in the PM, ES, and MF muscles between the DS group (PM, 1.5±0.3; ES, 1.7±0.4; MF, 1.1±0.2) and the non-DS group (PM, 1.4±0.3; ES, 1.7±0.5; MF, 1.2±0.3) (Table 2). In terms of the FI, as shown in Table 2, the PM muscle was significantly smaller in the DS group (0.11±0.08) than in the non-DS group (0.16±0.07) (p=0.031). The FI of the ES muscle was also significantly smaller in the DS group (0.18±0.09) than in the non-DS group (0.27±0.14) (p=0.010, Table 2). There were no significant differences in the FI of the MF muscle between the DS group (0.37±0.14) and the non-DS group (0.34±0.13). There were no significant differences in the vertebral CSA between the DS group (13.0±1.7) and the non-DS group (12.6±2.0, Table 2).

**Table 2:** FCSA index, GCSA index, FI of lumbar muscles, and vertebral CSA in the DS group and the non-DS group Data are presented as mean ± standard deviation. Asterisks (*) indicate statistically significant differences (p<0.05).

	DS	Non-DS	p-Value
FCSA index			
PM	1.3±0.3	1.2±0.3	0.16
ES	1.4±0.3	1.2±0.4	0.22
MF	0.7±0.2	0.8±0.2	0.27
GCSA index			
PM	1.5±0.3	1.4±0.3	0.59
ES	1.7±0.4	1.7±0.5	0.89
MF	1.1±0.2	1.2±0.3	0.65
FI			
PM	0.11±0.08	0.16±0.07	0.031*
ES	0.18±0.09	0.27±0.14	0.010*
MF	0.37±0.14	0.34±0.13	0.40
Vertebral CSA (cm^2^)	13.0±1.7	12.6±2.0	0.43
DS, degenerative spondylolisthesis; FCSA, functional cross-sectional area; non-DS, non-degenerative spondylolisthesis; PM, psoas major; ES, erector spinae; MF, multifidus; GCSA, gross cross-sectional area; FI, fat infiltration; CSA, cross-sectional area			

Correlation between the FCSA index, GCSA index, and FI of lumbar muscles, and DS

As shown in Table 2, there were no significant differences in the FCSA and GCSA indices of the lumbar muscles between the DS and non-DS groups. However, the DS group showed a significant trend toward a smaller FI of the PM and ES muscles than that of the non-DS group (Table 2). Therefore, multiple regression analyses evaluating correlations between the FI of the PM and ES muscles and DS were performed. As a result, there were no significant correlations between the FI of the PM muscle and the presence of DS (p=0.096, Table 3). However, the FI of the ES muscle significantly correlated with the presence of DS after adjustment for age, sex, scoliosis, LL, and SS (p=0.010) (standardized regression coefficient=-0.377; Table 3), indicating that the quality of ES muscle was better in the DS group than in the non-DS group.

**Table 3:** Multiple regression analyses evaluating correlations between dependent variables (FI of PM and FI of ES) and independent variables (presence of L4-DS) after adjustment for age, sex, scoliosis, LL, and SS Asterisk (*) indicates statistically significant differences (p<0.05).

Dependent variable	Independent variables	Regression coefficient	Standardized regression coefficient	t-Value	p-Value
FI of the PM muscle	L4-DS	-0.040	-0.243	-1.703	0.096
FI of the ES muscle	L4-DS	-0.093	-0.377	-2.667	0.010*
FI, fat infiltration; PM, psoas major; ES, erector spinae; LL, lumbar lordosis; SS, sacral slope; L4-DS, L4 degenerative spondylolisthesis					

Correlation between the FCSA index, GCSA index, FI of lumbar muscles, LL, and SS, and scoliosis

The correlation analyses revealed that the presence of scoliosis showed no significant correlation with the FCSA index, GCSA index, FI of lumbar muscles, LL, and SS after adjustment for age and sex.

Correlation between the FCSA index, GCSA index, or FI of lumbar muscles, and the lumbopelvic parameters in each group

In the DS group, there was no correlation between the FCSA, GCSA, and the FI of lumbar muscles, and the lumbopelvic parameters (LL and SS), except for a significant correlation between the GCSA index of the MF muscle and SS (p=0.04, Table 4). In the non-DS group, most of the CSA indices of the lumbar muscles did not show a significant correlation with the lumbopelvic parameters; however, the FCSA index of the ES and MF muscles and the GCSA index of the MF muscle showed a significant positive correlation with the lumbopelvic parameters (LL and SS) (Table 4).

**Table 4:** Correlation between the FCSA index, GCSA index, and FI of lumbar muscles, and the lumbopelvic parameters in each group Asterisks (*) indicate statistically significant differences (p<0.05).

Dependent variable	Independent variables		DS		Non-DS	
			Regression coefficient	p-Value	Regression coefficient	p-Value
LL	FCSA index	PM	-0.248	0.23	0.146	0.49
		ES	-0.033	0.88	0.420	0.037*
		MF	-0.059	0.78	0.575	0.0026*
	GCSA index	PM	-0.201	0.33	0.087	0.68
		ES	0.048	0.82	0.340	0.10
		MF	0.337	0.10	0.691	0.00013*
	FI	PM	0.189	0.37	0.173	0.41
		ES	0.084	0.69	-0.240	0.25
		MF	0.355	0.08	0.065	0.76
SS	FCSA index	PM	-0.143	0.49	0.217	0.30
		ES	0.102	0.63	0.477	0.016*
		MF	0.156	0.46	0.633	0.00068*
	GCSA index	PM	-0.088	0.68	0.188	0.37
		ES	0.152	0.47	0.297	0.15
		MF	0.415	0.04*	0.682	0.00017*
	FI	PM	0.142	0.50	-0.116	0.58
		ES	0.022	0.92	-0.374	0.07
		MF	0.182	0.38	-0.026	0.90
DS, degenerative spondylolisthesis; LL, lumbar lordosis; FCSA, functional cross-sectional area; non-DS, non-degenerative spondylolisthesis; SS, sacral slope; PM, psoas major; ES, erector spinae; MF, multifidus; GCSA, gross cross-sectional area; FI, fat infiltration						

## Discussion

In the patients who visited the hospital for reasons other than low back disorders, there were no significant differences in the FCSA and GCSA of the lumbar muscles in the evaluation of the quantity of lumbar muscles between patients with and without DS. Comparison of the FI of lumbar muscles, in which the quality of lumbar muscles is evaluated, showed that the FI of the PM and ES muscles was significantly smaller in patients with DS than in those without DS, suggesting that the quality of the PM and ES muscles is better in patients with DS. Further investigation is needed to clarify why different results were obtained between quantity and quality of the lumbar muscles. These results did not align with that of a previous report in which the MF muscle atrophy is commonly observed in patients with DS and is the primary cause of the DS. [19]. Other studies reported that LBP and adult spinal deformity correlated with lower CSA of the MF muscle and greater FI of the ES muscle [21,22]. Furthermore, a previous study reported that the CSA of the PM muscle was significantly decreased in the severe lumbar disability group compared with the mild/moderate disability group [23]. These findings suggest that patients with DS generally show an atrophic change of lumbar muscles. Previous studies reported that the PM and ES muscles have an important role in the maintenance of the lumbar lordotic angle [24,25]. Our finding that the quality of PM and ES muscles was better in patients with DS suggests that the function of the PM and ES muscles is to maintain the greater ULL angle in patients with DS. Considering that all the patients with DS in the present study had mild vertebral slip (grade I) and no patients had vertebral slip greater than grade II, we supposed that PM and ES muscles are strengthened in patients with mild vertebral slip and work to maintain LL, particularly ULL. In the author’s personal opinion, strengthening lumbar muscles may prevent the progression of DS and may be associated with maintaining LL in patients with DS, though it is unclear whether the improvement in muscle quality is the cause or result of vertebral slip.

With regard to lumbopelvic parameters, patients with DS exhibited a non-significant trend toward greater LL and significantly greater ULL. Previous studies reported that patients with DS showed significantly higher segmental LL at the upper lumbar spine, such as L1-L2 and L2-L3 levels, than patients without DS [26,27]. From these observations　[26,27], to maintain global sagittal alignment, the compensatory mechanism for the anterior translation of the L4 vertebral body may increase the degree of lordosis at the upper portion of the lumbar spine (L1-L4).

In patients without DS, the quantity of lumbar muscles, such as the ES and MF muscles, significantly correlated with the lumbopelvic parameters. However, in patients with DS, the quantity of the lumbar muscles, except the GCSA of the MF muscle, showed no correlation with the lumbopelvic parameters. Previous reports have shown that the CSA of the paraspinal muscle correlated with the lumbopelvic parameters [24,28]. In patients without DS, the quantity of the lumbar muscles significantly influenced the lumbopelvic parameters. However, in patients with DS, other factors, such as structural and degenerative factors, may be more correlated with lumbopelvic parameters than lumbar muscles.

We investigated the influence of spondylolysis on the quantities of the lumbar muscles and lumbopelvic parameters: PM atrophy is correlated with the progression of vertebral slip and greater LL and SS in patients with IS than without IS [25]. The results of the present study (patients with DS) differed from those of our previous study (patients with IS), regarding the correlation between the lumbopelvic parameters and the lumbar muscles, suggesting that difference in underlying pathomechanisms exists between DS and IS.

This study has several limitations. First, the number of patients was small. However, the patients included in the DS group were strictly limited to L4 level DS, and the patients in both groups were completely matched in terms of sex and age. Second, we evaluated the lumbopelvic parameters in the supine position and not in the standing position. These parameters necessarily change with the standing position. However, as mentioned previously, we believe that a CT study provides an advantage because more accurate measurements of lumbopelvic parameters can be obtained. We should understand that the clinical significance of our study may be different from studies evaluating lumbopelvic parameters in the standing position. Third, the degree of low back disorders in patients was not evaluated accurately. It may be overstated that the patients in this study were asymptomatic. We examined the patients who visited our hospital for reasons other than low back disorders. Thus, we should consider that our patient population was not completely equal to asymptomatic patients or general population.

## Conclusions

There was no difference in the quantity of lumbar muscles between patients with and without DS, but the quality of lumbar muscles (PM and ES) was better in patients with DS than in those without DS. Therefore, these findings indicate that the quality of lumbar muscles may be better in patients with mild DS than in those without DS. In addition, the quantity of lumbar muscles (ES and MF) was associated with the lumbopelvic parameters in patients without DS but not in those with DS. In conclusion, the strength of ES and MF is important to prevent the decrease of LL in non-DS patients, whereas only the strength of MF muscle may be associated with the maintenance of LL in DS patients.
